The article "Artificial Intelligence Analysis of EEG Amplitude in Intensive Heart Care" was published in 2021. Journal: J Healthc Eng.

# Artificial Intelligence Analysis of EEG Amplitude in Intensive Heart Care

**DOI:** 10.1155/2021/6284035

**Published:** 2021-07-02

**Authors:** Junjun Chen, Hong Pu, Dianrong Wang

**Affiliations:** Department of Intensive Care Unit, West China Hospital of Sichuan University, Chengdu 610041, China

## Abstract

This article first studied the morphological characteristics of the EEG for intensive cardiac care; that is, based on the analysis of the mechanism of disease diagnosis and treatment, a signal processing and machine learning model was constructed. Then, the methods of signal preprocessing, signal feature extraction, new neural network model structure, training mechanism, optimization algorithm, and efficiency are studied, and experimental verification is carried out for public data sets and clinical big data. Then, the principle of intensive cardiac monitoring, the mechanism of disease diagnosis, the types of arrhythmia, and the characteristics of the typical signal are studied, and the rhythm performance, individual variability, and neurophysiological basis of electrical signals in intensive cardiac monitoring are researched. Finally, the automatic signal recognition technology is studied. In order to improve the training speed and generalization ability, a multiclassification model based on Least Squares Twin Support Vector Machine (LS-TWIN-SVM) is proposed. The computational complexity of the classification model algorithm is compared, and intelligence is adopted. The optimization algorithm selects the parameters of the classifier and uses the EEG signal to simulate the model. Support Vector Machines and their improved algorithms have achieved the ultimum in shallow neural networks and have achieved good results in the classification and recognition of bioelectric signals. The LS-TWIN-SVM algorithm proposed in this paper has achieved good results in the classification and recognition of bioelectric signals. It can perform bioinformatics processing on intensive cardiac care EEG signals, systematically biometric information, diagnose diseases, the real-time detection, auxiliary diagnosis, and rehabilitation of patients.

## 1. Introduction

The biological body exhibits electrical changes during physiological activities, which are caused by the potential difference between the inside and outside of the corresponding cell membrane, which reflects the excitement changes of the corresponding parts, and is an important basis for biomedical clinical diagnosis. Bioelectric signals mainly include electrocardiogram (ECG), electroencephalogram (EEG), electrooculogram (EOG), and electromyogram (EMG) [1]. The bioelectric signal has the characteristics of small amplitude, low frequency, strong noise, and strong randomness, and has the characteristics of chaos, nonlinearity, and multichannel [2]. Therefore, useful signals are easily submerged in noise interference. For example, the ECG signal is in the order of mV, and the equipment collection must ensure the amplitude of 0.1–8 mV and the frequency range of 0.05–100 Hz. The amplitude of the ECG of a normal person is generally within 5 mV, and the energy is mainly concentrated in 0.5–45 Hz. The EEG signal is of the order of mV, and the frequency is below 60 Hz. The relative frequency of myoelectric and neuroelectric signals is relatively high, the frequency is 0–10 kHz, the amplitude of the myoelectric signal is below 5 mV, and the neuroelectric signal is of the order of mV [3]. The interference sources of bioelectric signal acquisition mainly include power frequency interference (50 Hz or 60 Hz), baseline drift, and interference from other components of biological signals [4]. Moreover, the signal is easily affected by the environment, psychology, and physiology and is a nonstationary random signal. The electrical signals are taken from the body surface, and the potential changes presented by different body surface positions are different. In order to detect the changes in the body surface potential in an all-round way, the measurement of bioelectric signals is often multichannel. For example, the standard ECG signal commonly used in clinical practice is 12 leads, while the EEG signal is 22 leads or more. Therefore, the processing methods of bioelectric signals are complex and diverse, and it is necessary to pay attention to signal processing algorithms that combine the time domain, frequency domain, and space domain [5]. Bioelectric signal recognition emphasizes robustness, accuracy, and repeatability, especially medical monitoring equipment, which requires real-time performance. Therefore, real-time effects must be considered on the premise of ensuring diagnostic accuracy. As the control center of the human body system, the brain directs various tissues, organs, and activities of the human body. The usual research methods for the brain include EEG, nuclear medicine imaging, MRI, cerebrovascular angiography, and other microscopic nerve detection method. Compared with other methods, EEG has the advantages of simple experiment, low cost, and relatively low requirements for the experimental environment. Therefore, from a practical point of view, EEG is very promising in brain research and the development of related products.

The article "Artificial Intelligence Analysis of EEG Amplitude in Intensive Heart Care" was published in 2021. Journal: J Healthc Eng.

Body surface physiological electrical signals such as ECG, EEG, and EMG have the characteristics of flexible collection; being noninvasive, economical, and convenient; and so forth and have been widely used in intelligent disease monitoring, diagnosis, and rehabilitation [6]. The characteristics of the bioelectric signal itself determine the complexity and diversity of its processing methods. The new intelligent auxiliary diagnosis and treatment system based on bioelectric signals integrates biomedicine, Internet technology, and artificial intelligence technology, and its processing process is a typical pattern recognition process. It generally consists of four parts: bioelectric signal acquisition, signal transmission and processing, intelligent identification, and information feedback or control [7]. The collection of bioelectric signals includes sensors and microprocessor units, which are responsible for signal collection, preliminary preprocessing, and format conversion. In the transmission stage, the signal is sent to the information center or the microprocessing unit, and then the signal filtering and other processing and intelligent auxiliary diagnosis are performed, and finally, the information is output or feedback to control the actuator. The key technology of intelligent auxiliary diagnosis system is signal processing and intelligent recognition algorithm, which determines the degree of intelligence and clinical application value.

With the development of advanced sensor technology and artificial intelligence technology, intelligent auxiliary diagnosis and treatment systems that integrate wearable devices, the Internet of Things, and wireless Internet have promoted pioneering changes in smart medicine. Auxiliary diagnosis and treatment technology based on bioelectrical signals started from the discovery of bioelectrical signals and experienced digitization and networking to the integration of the Internet of Things and wireless networks [7]. The corresponding collection equipment developed from digitization to portable and wearable, and the identification method of bioelectrical signals. It also includes advanced artificial intelligence algorithms from simple threshold judgment, statistical analysis.

This paper firstly studies the morphological characteristics of ECG and EEG signals, respectively; that is, based on the analysis of disease diagnosis and treatment mechanisms, it constructs signal processing and machine learning models and studies signal preprocessing, signal feature extraction methods, new neural network model structures, training mechanisms, and optimization algorithms and efficiency and for experimental verification of public data sets and clinical big data. In the second part, we study the principle of EEG in intensive cardiac care and the mechanism of disease diagnosis, the types of arrhythmia, and the characteristics of typical ECG; the rhythm performance, individual variability, and neurophysiological basis of EEG signals in intensive cardiac care are studied. The third part studies the signal automatic recognition technology. In order to improve the training speed and generalization ability, several multiclassification models based on the Least Squares Twin Support Vector Machine (LS-TWIN-SVM) are proposed, and the computational complexity of several model algorithms is compared. In addition, a variety of intelligent optimization algorithms are used to select the parameters of the classifier, and the EEG signal is used to simulate the model. Support Vector Machines and their improved algorithms have achieved the ultimate in shallow neural networks and good results in the classification and recognition of bioelectric signals.

The article "Artificial Intelligence Analysis of EEG Amplitude in Intensive Heart Care" was published in 2021. Journal: J Healthc Eng.

### 1.1. Analysis of Algorithm for Feature Extraction of ECG and EEG Signals

The bioelectric signal has the characteristics of multichannel and frequency band rhythm individual variability, and its feature extraction method involves multiple signal processing theories such as time domain, frequency domain, transform domain, and space domain [8].

### 1.2. ECG Signal Feature Extraction Method

The American Heart Association revised its opinions and was later promoted by the International Electrocardiology Society, forming a standard 12-lead ECG that is currently internationally recognized and used in various countries. According to the relationship of the ECG lead vector, the compression limb leads can also be derived from other leads. The standard 12-lead ECG includes limb leads I, II, III and compression limb leads VR, VL, and VF, and 6 chest leads V_l_, V_2_, V_3_, V_4_, V_5_, and V_6_; each lead reflects the different parts of the potential change. According to the theory of limb leads proposed by Einthoven, any limb lead can be deduced from the other two, namely, I + III = II. According to the relationship of the ECG lead vector, the compression limb leads can also be derived from other leads.

The feature extraction of the ECG signal is the key to guarantee the subsequent classification. The feature extraction method of the ECG signal can be divided into the direct extraction of the time domain waveform, the extraction of the frequency domain, or the feature extraction of the transform domain. The time-domain features are directly derived from the shape of the ECG waveform, which is more in line with the clinician's diagnostic habits. The time-domain features include the main wave amplitude, ST segment offset, QT interval, PP interval, RR interval, and RR interval ratio. Frequency domain features are signal values after frequency domain transformation, such as Discrete Fourier Transform (DFT) [9] and Power Spectral Density (PSD). Transform domain feature extraction is generally to extract the transform result or the coefficient of the transform domain function as the feature after the ECG signal is transformed in the transform domain, such as the statistics of the ECG signal [10], variance, discrete wavelet transform, wavelet packet decomposition, matching tracking algorithm, Hermite function, AR model parameters, and principal component analysis (PCA) [11]. The transform domain features do not need to rely on basic medical knowledge and the position information of each ECG wave but use mathematical methods to automatically analyze and calculate them, which is widely used in intelligent auxiliary diagnosis.

The article "Artificial Intelligence Analysis of EEG Amplitude in Intensive Heart Care" was published in 2021. Journal: J Healthc Eng.

### 1.3. Status of Intelligent Classification and Recognition Methods

According to the pattern characteristics of the ECG or EEG signal, it is the ultimate goal to complete automatic classification and recognition, explain the inner meaning reflected by the signal, and then output diagnostic information or control the actuator to perform auxiliary treatment [12]. The pattern classification methods of biological signals mainly include automatic knowledge modeling, statistical classification, traditional machine learning, and neural networks. The method of automatic knowledge modeling is based on knowledge expression and reasoning and is classified through logical reasoning according to the characteristic knowledge base such as signal shape, for example, fuzzy logic, expert system, and Markov model. This kind of method knowledge expression is intuitive and easy to understand, but it relies too much on knowledge expression; that is, it relies on expert experience, and the degree of intelligence is not high. Since the 1990s, statistical classification and machine learning techniques have gradually been used in biomedical signal classification, becoming the main branch of ECG and EEG signal classification methods. For example, Bayesian model (Bayes), K-Nearest Neighbor (KNN) [13], decision tree, and Linear Discriminant Analysis (LDA) [14]. Classical pattern classification methods have achieved certain results in the automatic identification of bioelectric signals, but the classification results and response speed are not satisfactory. With the development of neural network technology, especially deep learning technology in recent years, new breakthroughs have been made in biomedical assisted diagnosis. The following is a detailed analysis of the application status of neural network technology in the recognition of ECG and EEG signals.

The article "Artificial Intelligence Analysis of EEG Amplitude in Intensive Heart Care" was published in 2021. Journal: J Healthc Eng.

### 1.4. Traditional Neural Network Algorithm

In 1986, DE Rumelhart and GEHinton et al. proposed a neural network error backpropagation (EBP) [15] training algorithm, which solved the “exclusive OR” problem of the “perceptron” and reduced the neural network. After the 1990s, neural network methods have gradually been applied to the automatic classification and recognition of biological signals [16], and certain results have been achieved. Caricato et al. [17] proposed a neural network classification method based on the time characteristics of the EEG signal. Katheria et al. [18] extracted the time interval of the ECG signal, the high-order cumulant of the QRS complex, and other characteristics and used a fuzzy neural network to analyze the 7 types of ECG. The signal classification result reached 96%. Felze: et al. proposed a probabilistic neural network classification model for EEG signal classification and recognition. Das et al. [19] used modular neural networks to classify large-scale EEG signals and achieved good results. Dereymaeker et al. [20] used wavelet transform to extract features, and the accuracy of the classification of the four types of ECG signals by the multilayer perceptron network was 94%.

Traditional neural networks are difficult to find the optimal network structure and have limited fitting capabilities. In practical applications, in the face of data with large variability, the recognition accuracy fluctuates greatly, and the generalization ability is poor, which limits the clinical application of neural network automatic recognition technology.

### 1.5. Support Vector Machine and Its Extended Algorithm

Another popular and effective ECG and EEG signal classification algorithm is the Support Vector Machine. Support Vector Machine (SVM) is a supervised machine learning method proposed by Claessens et al. [21]. The algorithm is based on the minimum structural risk. The principle of transformation is to obtain the segmentation hyperplanes of different types of data and then classify and recognize the distance between the sample and the hyperplane. Claessens et al. proved that SVM can minimize the structural risk and is superior in the classification of small samples. The artificial neural network (ANN) method that can only minimize the empirical risk is flawed. Compared with traditional ANN, SVM has shown better generalization ability in solving small sample, nonlinear, and high-dimensional learning. Support Vector Machine, Least Squared Support Vector Machine (LS-SVM), and SVM combined with various intelligent optimization algorithms are widely used in the classification and recognition of EEG, ECG, and other biological signals. However, SVM needs to solve a large quadratic programming problem when solving the hyperplane. The increase in sample size leads to too much computational complexity, and the classification effect of SVM is not good when solving cross data.

The article "Artificial Intelligence Analysis of EEG Amplitude in Intensive Heart Care" was published in 2021. Journal: J Healthc Eng.

### 1.6. Analysis of the Diagnosis and Treatment Mechanism of ECG and EEG Signals

ECG is a technology that uses biosensor measuring electrodes to record the electrical activity pattern of the heart during each cardiac cycle from the body surface. It is one of the most commonly used examinations for clinical heart disease. It can not only help diagnose arrhythmia, myocardial ischemia, myocardial infarction, and location; evaluate the effect of drugs on the heart; monitor after cardiac surgery; determine the condition of pacemakers; and so forth but also be a must for routine surgical procedures and intensive care units (ICU).

### 1.7. Principles of Medical ECG

Electrical activation occurs when the heart is active. This electrical activation can cause changes in the body surface potential. According to the time sequence of cardiac activation, this body surface potential is recorded to form a continuous curve, which is called ECG. The abscissa of the standard ECG paper represents time, and each cell of 1 mm represents 0.04 s; the ordinate represents the amplitude, and each cell of 1 mm represents 0.1 mV.  Figure 1 shows the principle of the electrocardiogram. A complete EGG cycle includes atrial depolarization, ventricular depolarization, and ventricular repolarization. The complete cardiac process produces P wave, QRS complex wave, and T wave and PR interval, QT interval, and ST interval.

Several key interval indicators include the PR interval. The PR interval represents the time required for the excitement generated by the sinoatrial node to reach the ventricle through the atrium, the atrioventricular junction, and the atrioventricular bundle and causes the ventricle to start to excite; the QT interval is the time for the ventricular depolarization and repolarization process, which represents the heart. The ST segment represents that all parts of the ventricle have entered a depolarized state. At this time, there is no potential difference between the parts of the ventricle, so the ST segment curve is basically a horizontal state.

At present, the commonly used clinical ECG is 12-lead, which is called “standard lead.” The Dutch physiologist MacDarby et al. [22] proposed the concept of leads and the naming of ECG waveforms in 1903. In 1933, Wilson created unipolar limb leads VR, VL, and VF and precordial leads (thoracic leads) V1–V6, Akiyama et al. [23] modified the central electrical terminal and designed the compression limb leads. It is more practical and becomes the main body of clinical ECG.

The article "Artificial Intelligence Analysis of EEG Amplitude in Intensive Heart Care" was published in 2021. Journal: J Healthc Eng.

When the heart has arrhythmia or is damaged due to ischemia, or even necrosis, the changes in the electrical activity of the heart will be clearly reflected on the ECG, showing abnormal changes in the shape of each waveform; that is, the amplitude, shape, and time of the ECG signal features such as interval can reflect the underlying diseases of the heart and provide a reliable basis for doctors to diagnose various heart diseases. According to the standards of the American Association for the Advancement of Medical Devices (AAMD), more than a dozen common arrhythmias can be divided into 5 categories, namely, normal heartbeat (N, including normal heartbeat, left and right bundle branch block, etc.), supraventricular beats (S, including atrial premature beats, borderline premature beats, etc.), ventricular different beats (V, including ventricular premature beats and ventricular escape beats), ventricular fusion beats (F), and unknown beats (Q, pacing heartbeat, uncategorized heartbeat, etc.).  Figure 2 lists several common ECG signal time-domain waveforms of arrhythmia.

## 2. Experimental Design

### 2.1. Based on LS-TWSVM-Based Intensive Cardiac Monitoring EEG Amplitude Recognition

Scalp electrodes collect electroencephalogram (EEG) signals. This method has the characteristics of simple collection, noninvasiveness, high time resolution, low cost, convenience, and flexibility and is especially suitable for wearable systems. From the analysis in the first chapter, it can be seen that although advanced artificial intelligence technologies such as machine learning have greatly promoted the development of BCI technology of motor imagination, the current medical rehabilitation training system based on motor imagination BCI still has certain difficulties in its practical application. The main problems are that the accuracy of EEG source signals needs to be improved; the system response speed is limited; the recognition accuracy of EEG signals is not high; EEG sensorimotor rhythm is specific to different individuals, and even the same individual has greater variability at different times and different physical conditions.

In response to the existing problems, this chapter proposes an EEG motion image signal recognition algorithm based on adaptive frequency band selection CPS feature extraction combined with Least Squares Twin Support Vector Machine (LS-TWIN-SVM) classification. First, use adaptive artifact removal technology to filter the signal to improve the accuracy of the EEG signal, then use a band-pass filter to generate EEG rhythm signals of different frequency bands, perform CSP feature extraction, and finally send it to the LS-TWIN-SVM classifier for adaptive selection. In the optimal frequency band, the classifiers select the frequency band characteristics for a specific person and perform real-time recognition. In order to improve the accuracy of EEG signal recognition, various kernel functions were tested, and several biointelligence optimization algorithms were compared to select the optimal classifier parameters. The public data set is used as the test object to verify the feasibility of the proposed algorithm. The following sections will explain in detail.

The article "Artificial Intelligence Analysis of EEG Amplitude in Intensive Heart Care" was published in 2021. Journal: J Healthc Eng.

### 2.2. Least Squares Twin Support Vector Machine (LS-TWIN-SVM) Algorithm Modeling

Support Vector Machine (SVM) classification seeks an optimal hyperplane based on the principle of structural risk minimization, which maximizes the blank area on both sides of the hyperplane while ensuring the accuracy of the training sample classification. For the linear case, as shown in Figure 3, the straight line *H* is a dividing line with *W* as the normal vector. This dividing line can divide the two types of data as accurately as possible. *H*_1_ and *H* are the two types of samples. The support vector points and the straight line parallel to the classification line are analyzed. When *H* is in the middle of *H*_1_ and *H*_2_, the line meets the principle of maximizing the interval between the two types of sample points and becomes the optimal dividing line. This is converted to the problem of finding the normal vector. Extending to a high-dimensional space, the optimal classification line becomes the optimal hyperplane, that is, finding the normal vector of the optimal classification hyperplane and classifying multiclass samples by finding the distance.

Taking the two-classification problem as an example, given the training sample set (*α*_*i*_, *β*_*i*_)*i*=1,2,…, *n*, *α* ∈ *R*^*n*^, *β* ∈ {±1} of the two types of data, the hyperplane is analyzed. If the sample is correctly classified and the classification interval is as large as possible, the hyperplane must satisfy the following constraints:

(1) $$\begin{array}{c} \left\{\begin{array}{cc} w\alpha_{i}+b\geq \beta_{i} & \beta_{i}=+1,\\ w\alpha_{i}+b\leq \beta_{i} & \beta_{i}=-1. \end{array}\right) \end{array}$$

When combined, they can be expressed as follows:

(2) $$\begin{array}{c} w\alpha_{i}+b\geq \frac{1}{\beta_{i}},\;i=1,2,...,n. \end{array}$$

Then, the classification interval can be expressed as follows:

(3) $$\begin{array}{c} \min\left\{\frac{\left(w\alpha_{i}+b\right)}{\left\|w\right\|}\right\}=\frac{2}{\left\|w\right\|}+\max\left\{\frac{\left(w\alpha_{i}+b\right)}{\left||w|\right|}\right\}. \end{array}$$

Therefore, the goal of SVM is to maximize the classification interval under the condition of satisfying the constraint formula (2), that is, to solve the problem of the following formula [24]:

(4) $$\begin{array}{c} \min f\left(w\right)=\frac{1}{2{\left\|w\right\|}^{2}}=\frac{1}{2}\left(w^{T}w\right). \end{array}$$

When there is a linear inseparable pattern, the optimal segmentation hyperplane is required to meet the principle of minimum average classification error probability for all training samples. At this time, just relax the constraint condition of formula (2), that is, introduce a slack variable *ξ*_*i*_; then, formula (2) becomes

(5) $$\begin{array}{c} w\alpha_{i}+b\geq \frac{\left(1-\xi_{i}\right)}{\beta_{i}},\;i=1,2,\ldots ,n. \end{array}$$

To introduce a cost function into the objective function, that is, add a penalty component with an adjustable factor *λ* to function (4), the objective function formula (4) can be expressed as

(6) $$\begin{array}{c} \min f\left(w\right)=\frac{1}{2{\left\|w\right\|}^{2}}+\lambda \sum_{i=1}^{n}\xi_{i}\\ =\frac{1}{2\left(w^{T}w\right)}+\lambda \sum_{i=1}^{n}\xi_{i}. \end{array}$$

Among them, *λ* is the penalty factor, which controls the degree of punishment for the wrong sample. The larger *ξ*_*i*_, the heavier the penalty for the error.

The article "Artificial Intelligence Analysis of EEG Amplitude in Intensive Heart Care" was published in 2021. Journal: J Healthc Eng.

### 2.3. Twin Support Vector Machine

Support Vector Machines show strong generalization and promotion capabilities in small sample and nonlinear classification problems. However, there are still some challenges. For example, when facing a large sample, the optimal solution can be obtained by solving a large-scale quadratic programming problem. The training speed is slow and it is difficult to meet certain real-time systems. In addition, SVM is not very suitable for processing cross-type data.

Twin Support Vector Machine (TWSVM) is proposed on the basis of generalized eigenvalue proximal SVM (GEPSVM). As shown in Figure 3, for the binary classification problem, TWSVM constructs an optimal near-end hyperplane for each class. By solving two small quadratic programming problems, such sample points are “close” to the hyperplane, and the other sample point is appropriately far away from the hyperplane [25]. Compared with traditional Support Vector Machines, the learning efficiency is improved.

## 3. Results and Analysis

### 3.1. Comparison of EEG Signal Classification Results of Twin Support Vector Machine and Its Extended Algorithm

The genetic algorithm (GA) and quantum genetic algorithm (QGA) are widely used algorithms. The genetic algorithm is a biological incentive algorithm, which has been successfully used to solve engineering problems such as complex optimization and feature extraction. Good results have been achieved in the multiparameter optimization selection problem. The genetic algorithm's parameter search process for the classifier is as follows:

1. Population initialization and parameter coding.
2. Calculate the fitness function of each chromosome.
3. Use GA calculation steps: selection, crossover, and mutation.
4. The offspring replace the old population to form a new population of the next generation.
5. Obtain the classifier parameter model. When the iterative conditions are met, the optimal chromosome is generated; otherwise, it returns to step 2.

The article "Artificial Intelligence Analysis of EEG Amplitude in Intensive Heart Care" was published in 2021. Journal: J Healthc Eng.

The implementation process of quantum genetic algorithm is based on the basic framework of genetic algorithm, adding concepts such as quantum states and quantum gates in quantum theory and using qubits and superposition states to encode chromosomes [26]. The typical iterative process of QGA includes selection, mutation operation (quantum crossover, quantum mutation, and quantum interference), quantum measurement, evaluation, and substitution.

### 3.2. EEG Signal Recognition of the LS-TWIN-SVM Classifier Based on Intelligent Optimization Algorithm

The biological intelligence optimization algorithm and its improved algorithm have been successfully used in the parameter adjustment of the neural network classifier, but the convergence and final performance are greatly affected by the classifier and the data set. This section uses PSO, CPSO, GA, and QGA algorithms to test the proposed classifier models, respectively. In order to achieve higher efficiency and optimal classification results, the CPU running time, classifier training, and testing of several optimization algorithms are compared.

The maximum iteration algebra of the four optimization algorithms is set to 300, and the optimal classification accuracy rate of 10-cv cross-validation on the training data set is used as the fitness function. The population size is 40, the individual length is 20, and the genetic algorithm generation gap is set to 0.95. The crossover and mutation probabilities are set to 0.7 and 0.01, respectively. Quantum genetic algorithm combines the principles of genetic algorithm and quantum mechanics. The process includes initializing population and coding classifier parameters, calculating fitness function, selection, mutation, evaluation, and replacement. The mutation operation of the evolutionary algorithm uses the quantum revolving door strategy. For the convenience of comparison, the population size and individual length of QGA are the same as the GA algorithm settings, and the quantum rotation angle is set to 0.01.

The parameters of the particle swarm optimization (PSO) algorithm are set as follows: the population size is 20, and the acceleration constants are set to 1.5 and 1.70, respectively. During the implementation of the chaotic particle swarm optimization (CPSO) algorithm, two chaotic sequences are generated to prevent the PSO algorithm from falling into the local maximum. In the initialization phase, chaotic initialization is used to select the initialization position instead of random selection; in the optimization position selection process, the global optimization position obtained by the particle search is subjected to chaos operation, and then the particle position is determined by the global optimization position after the chaos operation. The CPSO parameter settings are the same as PSO, and the parameters can be randomly generated.

The article "Artificial Intelligence Analysis of EEG Amplitude in Intensive Heart Care" was published in 2021. Journal: J Healthc Eng.

Use the CSP features extracted from the data set to test the classifier algorithm. The experimental results are shown in Figures 4 and 5. As can be seen from the figure, the test results of the data set show that the classification effect of the classifier based on PSO and GA is equivalent, and the accuracy is better than the CPSO and QGA algorithms. However, in the test results of the second data set, the PSO and CPSO algorithms are significantly better than the GA and QGA parameter optimization results. From Figure 6, it is obvious that PSO has the highest operating efficiency and simple calculation, which is convenient for real-time hardware implementation. Therefore, TWIN-SVM is chosen as the classifier of the MI-BCI system.

### 3.3. Analysis of Experimental Results

Since its introduction, TWIN-SVM has been successfully applied in many fields, and scholars have made a lot of contributions to the algorithm expansion and application of Twin Support Vector Machines, and it has also been successfully used in the intelligent recognition of biomedical signals.

In order to improve the system response speed and overcome the variability of individual EEG rhythms, this chapter proposes adaptive artifact removal and adaptive frequency band selection feature extraction methods to enhance the classification and recognition of EEG signals. And the TWIN-SVM classifier is used for the rapid classification and recognition of EEG. Experimental results are shown in Table 1, which showed that the classification accuracy rate, CPU operating efficiency, and other indicators have been significantly improved.

The proposed TWIN-SVM method shows good results on the data set as shown in Figure 7. The proposed method performs adaptive frequency band selection, which overcomes the frequency band variability of EEG signals between individuals. However, as can be seen from Figure 8, the optimal cross-validation accuracy rate on the training data set and the test accuracy rate on the test data set are quite different, indicating that the data at different test times has greater variability; that is, there is still variability within the individual. We should conduct more EEG experiments. The more samples are in the experiment, the closer the results are to the essence of the facts. The experiment reported in this article can be said to be a preliminary exploration of EEG experiments under different conditions. The next step is to carry out more experiments: one is to increase the samples of existing experiments and the other is to expand the experimental projects and conduct experiments on more states.

The article "Artificial Intelligence Analysis of EEG Amplitude in Intensive Heart Care" was published in 2021. Journal: J Healthc Eng.

## 4. Conclusion

EEG is combined with more analysis methods to analyze the activities of various parts of the brain. EEG has its irreplaceable advantages, but it also has its disadvantages. If it can be combined with other suitable methods and learn from each other's strengths, the completeness and persuasiveness of the experiment can be further strengthened, for example, using EEG combined with functional imaging techniques such as PET and magnetoencephalography. The machine learning method is a powerful tool for the recognition of EEG signals in intensive cardiac care, and many achievements have been made in this field. However, the rehabilitation system based on EEG still has not achieved large-scale clinical application. The main reason is that the technology still has the following problems: firstly, there is great variability for different individuals based on the amplitude of EEG, and even the same individual at different times. There are also differences with the environment, which requires the system to have stronger adaptability; secondly, there is a lot of interference in the scalp EEG signal, and the signal source accuracy is limited, which affects the recognition accuracy; finally, more efficient adaptation is needed. Aiming at the above problems, this paper proposes adaptive artifact removal theory, adaptive frequency band selection feature extraction, and a fast TWIN-SVM classification strategy based on PSO. In order to evaluate the effect of this method, a classifier model based on a kernel function and an intelligent optimization algorithm is used to optimize the classifier. Neuroinformatics is a newly emerging interdisciplinary subject. It is still in its infancy, and there is still a big gap with the established goals. Although EEG has existed for a long time, due to the complexity of the EEG signal itself, much of the information still cannot be extracted. With the development of signal processing methods, more and more simple and efficient data processing methods have been developed. This has greatly promoted the development and application of EEG in neuroinformatics. Through the study of EEG, it can further help to understand how the human brain works in different modes and promote the development of neuroinformatics.

The article "Artificial Intelligence Analysis of EEG Amplitude in Intensive Heart Care" was published in 2021. Journal: J Healthc Eng.

## Figures and Tables

**Figure 1:** ECG single heartbeat waveform.

**Figure 2:** Several types of arrhythmia heartbeat signals.

**Figure 3:** Twin Support Vector Machine two-dimensional data classification diagram.

**Figure 4:** The classification effect of the first data set optimization algorithm.

**Figure 5:** The classification effect of the second data set optimization algorithm.

**Figure 6:** Comparison of running time of the optimized method.

**Figure 7:** Comparison between PSO-LS-TWIN-SVM and common recognition algorithms.

**Figure 8:** The average and standard error of recognition algorithms.

**Table 1:** TWIN-SVM and common recognition algorithms results.

Testing objects	PSO-LS-TWIN-SVM	LDA	BP	PNN
1	88.19	87.24	72.43	83.45
2	64.35	57.32	62.34	61.35
3	93.42	91.34	97.53	88.24
4	65.34	63.24	71.34	70.12
5	76.35	54.87	52.34	50.35
6	67.34	70.23	74.45	65.24
7	75.23	70.43	74.14	58.33
8	88.89	83.25	87.24	91.34
9	78.34	73.42	76.35	73.24
10	67.24	70.78	66.24	70.43
Mean	76.47	72.21	73.44	71.21
SE	11.24	13.34	12.32	16.31

## Data Availability

Data are available from the corresponding author upon request.
